RETRACTED

# Down-regulation of miR-133a and miR-539 are associated with unfavorable prognosis in patients suffering from osteosarcoma

**DOI:** 10.1186/s12935-015-0237-6

**Published:** 2015-09-17

**Authors:** Alireza Mirghasemi, Afshin Taheriazam, Seyyed Hasan Karbasy, Ali Torkaman, Mohammadreza Shakeri, Emad Yahaghi, Aram Mokarizadeh

**Affiliations:** Department of Orthopedics, Qom University of Medical Sciences, Qom, Iran; Department of Orthopedics Surgery, Tehran Medical Sciences Branch, Islamic Azad University, Tehran, Iran; Department of Anesthesiology, Birjand University of Medical Sciences, Birjand, Iran; Department of Orthopedics, Firoozgar Hospital, Iran University of Medical Sciences, Tehran, Iran; Department of Orthopaedic and Trauma Surgery, Birjand University of Medical Sciences, Birjand, Iran; Department of Molecular Biology, Baqiyatallah University of Medical Sciences, Tehran, Iran; Cellular & Molecular Research Center, Kurdistan University of Medical Sciences, Sanandaj, Iran

**Keywords:** MicRNA, Survival, Patient, Marker, Cancer

## Abstract

**Background:**

MicroRNAs (miRNAs) play key roles in cancer development and progression. The purpose of the present study was to determine the expression levels of miR-133a and miR-539 in osteosarcoma patients and to further investigate the clinicopathological, and prognostic value of these miRNAs.

**Methods:**

The expression levels of miR-133a and miR-539 were determined by qRT-PCR. Associations between miRNAs expressions and various clinicopathological characteristics were analyzed. Survival rate was determined with Kaplan–Meier and statistically analyzed with the log-rank method between groups. Survival data were evaluated through multivariate Cox regression analysis

**Results:**

Our findings revealed that the miR-133a expression was significantly decreased in clinical osteosarcoma tissues compared to adjacent normal bone tissues. The expression level of miR-539 was decreased in clinical osteosarcoma tissues as compared to those adjacent normal tissues. Low expressions of miR-133a and miR-539 were significantly association with advanced TNM stage (P = 0.002; P = 0.001), and metastasis or recurrence (P = 0.001; P = 0.01). Furthermore, Kaplan–Meier survival analysis and log-rank test showed that the low expressions of miR-133a and miR-539 were correlated with the reduced overall survival of osteosarcoma patients. Multivariate Cox proportional hazards model showed that decreased expressions of miR-133a and miR-539 (P = 0.007; P = 0.02), TNM stage (P = 0.001; P = 0.002), and metastasis or recurrence (P = 0.005; P = 0.026) were independent prognostic markers of overall survival of patients.

**Conclusion:**

These results suggest that decreased miR-133a and miR-539 expressions may participate in the progression of osteosarcoma. Together, these results showed that miR-133a and miR-539 may have their role in both progression and prognosis of osteosarcoma.

RETRACTED

## Background

One of the most common primary bone tumors in children and adolescents is osteosarcoma, which is most often localized in the metaphysis of the adolescent long bones [1]. More than 50 % of patients who are chemoresistant have an extremely poor prognosis due to lung metastasis [2]. The 5-year overall and disease-free survival rates for osteosarcoma patients are around 50–60 % [3]. Despite the advances in therapeutic strategies, there is dissatisfactory for most osteosarcoma patients with metastasis or recurrence. Therefore, it is required to identify biomarkers, and therapeutic targets for osteosarcoma.

MicroRNAs (miRNAs) are endogenous 19e25 nt noncoding RNAs that can bind the 3′-untranslated region (3′-UTR) of specific genes to inhibit the translation of corresponding mRNA targets. Increasing evidence demonstrates that the deregulations of miRNAs are involved in various biological processes including proliferation, differentiation, and apoptosis [4]. Current evidences indicate that miRNAs have their role in tumorigenesis and provide new insights into the molecular mechanisms underlying carcinogenesis. Different miRNAs have been shown to participate in the initiation and progression of osteosarcoma [5–8]. Recently, it has been reported that miR-539 may inhibit cell proliferation through suppressing the MITF expression [9]. MiR-539 were confirmed to be down-regulated in osteosarcoma cell lines [10, 11]. MiR-133a is also shown to be an important regulator in osteogenesis, and its down-regulation has been reported in bone morphogenetic protein (BMP)-induced osteogenesis. Moreover, it can function as suppressor of RunX2 expression for inhibition of osteoblast differentiation [12]. Further investigations are required to identify miR-133a and miR-539 expression levels in clinical osteosarcoma patients and its potential roles in osteosarcoma carcinogenesis and progression. Therefore, we examined the clinical importance of miR-133a and miR-539 expressions in osteosarcoma tissue samples using real-time PCR.

## Methods

### Patients

The samples of cancer tissue and corresponding noncancerous bone tissues were collected between 2010 and 2014 from 35 patients who were undergoing surgery in different hospitals of Tehran, Iran. None of the patients received radiotherapy and chemotherapy before the tissues were collected. Informed consents were obtained from all the patients. All specimens were obtained during surgery, frozen immediately in liquid nitrogen, and were stored at -80 °C. Furthermore, the diagnosis and the histological grading were proved by pathologists. The clinicopathological features are summarized in Tables 1 and 2.

RETRACTED

**Table 1:** The association between miR-133a expression and characteristics of patients suffering from osteosarcoma

Clinicopathological features	No. of cases	Expression of miR-133a		*P* value of miR-133a
		Low, 19	High, 16	
Gender				
Male	18	6	12	NS
Female	17	13	4	
Age				
≤40	20	9	11	NS
>40	15	10	5	
Tumor diameter (cm)				
≤5	21	10	11	NS
>5	14	9	5	
Differentiation				
Well and moderate	16	7	9	NS
Poor	19	12	7	
TNM stage				
I + II	15	5	10	0.002
III + IV	20	14	6	
Metastasis or recurrence				
Yes	19	16	3	0.001
No	16	3	13

**Table 2:** The association between miR-539 expression and characteristics of patients suffering from osteosarcoma

Clinicopathological features	No. of cases, 35	Expression of miR-539		*P* value
		Low, 21	High, 14	
Gender				
Male	15	9	6	NS
Female	20	12	8	
Age				
≤40	19	10	9	NS
>40	16	11	5	
Tumor diameter (cm)				
≤5	21	11	10	NS
>5	14	10	4	
Differentiation				
Well and moderate	18	9	9	NS
Poor	17	12	5	
TNM stage				
I + II	12	5	7	0.001
III + IV	23	16	7	
Metastasis or recurrence				
Yes	22	16	6	0.01
No	13	5	8	

### Real-time quantitative PCR

Total RNA was extracted using miRNeasy kit (Qiagen) according to the manufacturer’s instructions. The expression levels of miRNAs quantitated using the TaqMan miRNA assey kit (Applied Biosystems). Real-timePCR was performed using Rotor Gene 6000 Real-Time PCR (Qiagen, Germany) with an invitrogen kit and a TaqMan universal PCR master mix. The relative expression levels of miRNAs were normalized to that of internal control U6 by using $2^{{ - \Delta \Delta {\text{C}}_{\text{t}} }}$ cycle threshold method [13].

### Statistical analysis

Our data were evaluated using SPSS 19.0 software (SPSS Inc., USA). The differences between two groups were analyzed using the Student’s t-test. The statistical analysis of cases in groups were performed using the Chi square test. Moreover, log-rank test and Kaplan–Meier method were used to evaluate survival rate in patients with osteosarcoma. Multivariate analysis was performed to evaluate prognostic values using Cox proportional hazards model. P < 0.05 was used to indicate a statistically significant difference.

## Results

As demonstrated by quantitative real-time PCR, the miR-133a expression was significantly decreased in clinical osteosarcoma tissues (median relative expression level ± SD: 3.74 ± 1.83) compared to adjacent normal bone tissues (median relative expression level ± SD: 15.23 ± 3.25, P < 0.001; Fig. 1).

**Fig. 1:** The relative expression level of miR-133a between osteosarcoma bone tissue and noncancerous bone tissues

The expression level of miR-539 was decreased in clinical osteosarcoma tissues (median relative expression level ± SD: 2.23 ± 1.02) as compared to that adjacent normal tissues (mean ± SD: 5.68 ± 1.42, P < 0.0001; Fig. 2).

RETRACTED

**Fig. 2:** The relative expression level of miR-539 between osteosarcoma bone tissue and noncancerous bone tissues

### Correlation of miRNAs expressions with the clinicopathological fetures

The patients with osteosarcoma were classified into two groups based on the median expression levels.

Low expression of miR-133a showed significant association with advanced TNM stage (P = 0.002), and metastasis or recurrence (P = 0.001). But no significant association with other clinical factors (Table 1). On the other hand, low expression of miR-539 were significantly correlated with advanced TNM stage (P = 0.001), and metastasis or recurrence (P = 0.01). But no significant association with other clinical factors (Table 2). Furthermore, Kaplan–Meier survival analysis and log-rank test showed that the low expressions of miR-133a and miR-539 were correlated with the reduced overall survival of osteosarcoma patients (log-rank test P < 0.001; Figs. 3, 4). Multivariate Cox proportional hazards model showed that decreased expressions of miR-133a and miR-539 (P = 0.007; P = 0.02), TNM stage (P = 0.001; P = 0.002), and metastasis or recurrence (P = 0.005; P = 0.026) were independent prognostic markers of overall survival of patients (Tables 3, 4).

**Fig. 3:** Correlation between miR-133a expression and survival in patients

**Fig. 4:** Correlation between miR-539 expression and survival in patients

**Table 3:** Multivariate analysis of the correlation of prognosis miR-133a with clinicopathological factors

Clinicopathological characteristics	HR	95 % CI	*P* value
Gender	1.264	0.624–1.612	0.521
Age	1.365	0.725–1.937	0.4
TNM stage	3.618	1.319–10.261	0.001
Tumor diameter (cm)	0.89	0.615–1.523	0.2
Metastasis or recurrence	3.28	3.278–9.972	0.005
Differentiation	1.015	0.693–1.371	0.31
miR-133a expression	3.421	1.326–9.371	0.007

**Table 4:** Multivariate analysis of the correlation of prognosis miR-539 with clinicopathological factors

Clinicopathological characteristics	HR	95 % CI	*P* value
Gender	1.03	0.532–1.762	0.541
Age	0.73	0.382–1.108	0.527
TNM stage	4.96	2.462–11.72	0.002
Tumor diameter (cm)	1.21	0.73–2.03	0.374
Metastasis or recurrence	3.77	1.538–8.725	0.026
Differentiation	1.316	1.035–2.441	0.3
miR-539 expression	3.68	2.153–10.227	0.02

## Discussion

Various deregulated miRNAs, have been reported in osteosarcoma development [14]. Nevertheless, it is still an ongoing process to elucidate new important deregulated miRNAs and their roles in cancer carcinogenesis and progression. In the present study, we found that the miR-133a was significantly decreased in clinical osteosarcoma tissues compared to adjacent normal bone. Moreover, low expression of miR-133a showed significant association with advanced TNM stage, and metastasis or recurrence. Kaplan–Meier survival analysis and log-rank test showed that the low expression of miR-133a was correlated with the reduced overall survival of osteosarcoma patients. Multivariate Cox proportional hazards model showed that decreased expressions of miR-133a, TNM stage, and metastasis were independent prognostic markers of overall survival of patients. Recently, miR-133a is also reported to be an important regulator in osteogenesis, and miR-133a expression was proved to play an important role during osteoblast differentiation, by the finding that BMP2 treatment could decrease the expression of miR-133a during osteoblast lineage commitment and osteogenesis [12]. Ji et al. [15] reported that miR-133a expression was significantly suppressed in tumor tissues as compared to that in adjacent normal tissues. They found that miR-133a expression in tumor tissues was significantly reverse-correlated with osteosarcoma clinical tumor and Kaplan–Meier survival analysis also revealed that low miR-133a expression in tumor tissues was significantly correlated with the reduced overall survival of osteosarcoma patients.

RETRACTED

They indicated that miR-133a might function as a tumor suppressor or an antionco-miRNA in cancer carcinogenesis and progression. Previous reports revealed the roles of miR-133a in some other kinds of cancer, such as prostate cancer, bladder cancer, and esophagus cancer [16–18]. Among them, miR-133a expression is down-regulated in all these types of cancer, but the underlying mechanisms which mediate the down-regulation of miR-133a in cancer required to further investigations.

Previous studies reported that the expression of Bcl-xL, is also associated with overall survival of osteosarcoma patients [19]. These results indicated that miR-133a may be effective to predict the prognosis of osteosarcoma patients. Human important anti-apoptotic molecules Bcl-xL and Mcl-1 are determined to be new direct targets of miR-133a in osteosarcoma, indicating that miR-133a may exert its pro-apoptotic function throughout inhibiting Bcl-xL and Mcl-1 expression. Human EGFR, TAGLN2, and FSCN1 reported to be molecular targets of miR-133a in other kinds of cancers [16–18]. The recent evidence indicated that cancer pathways may be regulated by miR-133a expression, and miR-133a may be a new therapeutic target to repress cancer progression.

RETRACTED

In the present study, the expression level of miR-539 was decreased in clinical osteosarcoma tissues as compared to those adjacent normal tissues. Furthermore, low expression of miR-539 was significantly correlated with advanced TNM stage, and metastasis or recurrence. Kaplan–Meier survival analysis and log-rank test showed that the low expression of miR-539 was correlated with the reduced overall survival of osteosarcoma patients. Multivariate Cox proportional hazards model showed that decreased expressions of miR-539, TNM stage, and metastasis or recurrence were independent prognostic markers of overall survival of patients. Recently, it has been reported that miR-539 may inhibit cell proliferation through suppressing the MITF expression [9]. Moreover, miR-539 were confirmed to be down-regulated in osteosarcoma cell lines [10, 11].

There are few studies that have described the function of miR-539. One study indicated that miR-539 is among the factors sensing cellular biotin levels and targets holocarboxylase synthetase (HCS) [12]. Another study, showed that miR-539 suppress *O*-GlcNAcase expression and play an important role in the failing heart [20]. Moreover, it has been reported that miR-539 participates in the regulation of mitochondrial activity and apoptosis through targeting PHB2 [21].

The expression of miR-539 was previously analyzed in human thyroid cancer cell lines and in normal thyroids (NT). It has revealed that miR-539 expression was decreased compared to normal control [22]. Furthermore, it has been found that miR-539 plays a suppressor role in thyroid cancer cell migration and invasion and miR-539 binding to the 3′-UTR region of CARMA1 inhibited the expression of CARMA1 in thyroid cancer cells. Mentioned study indicated that miR-539 is a novel regulator of migration and invasion in human thyroid cancer cells by targeting CARMA1 [22]. However, further studies are needed to verify the role miR-539 in developing of different cancer types.

## Conclusion

In conclusion, these results suggest that decreased miR-133a and miR-539 expressions may participate in the progression of osteosarcoma. Together, these results showed that miR-133a and miR-539 may have their role in both progression and prognosis of osteosarcoma. However, further studies are required to identify the role of these miRNAs in progression and prognosis of osteosarcoma by their targets.
